This article has been retracted.

# Association between Interleukin-4-590C>T Polymorphism and the Susceptibility to Asthma: A Meta-Analysis of Case-Control Study

**DOI:** 10.1155/2022/1712715

**Published:** 2022-03-29

**Authors:** Tong Liu, Weimou Yin, Ling Luo, Yankui Wu, Songmei Qin, Xuejun Qin

**Affiliations:** Department of Respiratory Medicine, The People's Hospital of Guangxi Zhuang Autonomous Region, Nanning, China

## Abstract

This study was aimed to investigate the relationship between the interleukin-4-590C > T gene polymorphism and the susceptibility to asthma by meta-analysis. To explore the underlying relationship between the polymorphism of IL-4-590C > T and the susceptibility to asthma, this study systematically retrieved the literature including cohort studies and case-control studies published before June 2019 in PubMed, Embase, and Cochrane Library. Data on the odds ratio (OR) and 95% confidence interval (CI) of the literature were included in the relative studies. Subsequently, the included data were weighted by an inverse variance and then analyzed by the fixed or random effects model. Overall, 818 asthma patients and 831 healthy individuals participated in the 8 independent case-control studies in the current meta-analysis. There was no correlation between IL-4-590C > T TT genotype and the increased susceptibility to asthma (dominant model: OR = 1.31, 95% CI = 0.68–2.53). Subgroup analysis by ethnicity showed no significant results in the Asians (OR = 1.28, 95% CI = 0.24–6.80); however, IL-4-590C > T TT genotype significantly elevated the susceptibility to asthma in the Caucasians (OR = 1.43, 95%CI = 1.03–1.98). Meanwhile, subgroup analysis was performed by source of control. A statistically significant result was found in the population-based control group (OR = 1.33, 95% CI = 1.01–1.76), but not in the hospital-based control group (OR = 1.22, 95% CI = 0.27–5.46). The results demonstrated that IL-4-590C > T TT genotype could significantly enhance the susceptibility to asthma in Caucasians without increasing that in Asian populations. However, it still required a large sample of high-quality studies in multicentral hospital to further confirm its reliability.

## 1. Introduction

Bronchial asthma, referred to as asthma, is a chronic inflammation of the airway characterized by increased airway reactivity, reversible airflow limitation, and increased mucosal secretion. There are many types of cells involved in its development, such as mast cells, eosinophils and T-lymphocyte infiltration, and many other inflammatory cells and cellular components [1–3]. In recent years, with the improvement of people's living standards and the gradual deterioration of living environment, more and more people, especially children, are diagnosed with asthma [4]. The incidence of asthma varies between different regions and countries. Generally, in developed countries and urban areas where economic development is relatively fast, environmental pollution and other factors have led to higher incidence compared with developing countries [5]. Numerous studies have shown that environmental factors could cause asthma symptoms by affecting the patient's gene expression, which in turn affected its immune response to various inhalants [6–8].

Nowadays, most researchers have more and more in-depth introduction and understanding on the difficulty and severity of asthma-related genes and its gene polymorphisms, which resulted into becoming hot issues [9, 10]. Previous studies on related genes have produced different results, which have met an agreement that asthma was a complex genetic disease involving multiple genes and chromosomal regions' mutations [11, 12]. In addition, interleukin-4 (IL-4) gene has attracted much attention, In addition, interleukin-4 (IL-4) gene, located on the same chromosome (5q3l-q33 and 5q23-31, respectively), has attracted much attention in recent years, and its transcribed cytokines have some of the same structure and function [13, 14]. A large number of polymorphic sites in the IL-4 genome have been reported, and the susceptibility to asthma are associated with reported polymorphisms [15, 16]. Many investigations have conducted a series of clinical studies on whether the mutation at a certain site of the IL-4 gene increased the probability of asthma in children, and the results were not the same [17]. Here, we analyzed the polymorphism of IL-4-590C/T gene through obtaining relevant genetic characteristic data and exploring the relationship between mutations at the IL-4 gene locus and the risk of asthma. We explored whether the IL-4 gene had a synergistic effect in the pathogenesis of asthma, thus discussing the pathogenesis of asthma from a genetic perspective and providing a premise for the prevention and diagnosis of the disease, and lay the foundation for preventing and reducing adult asthma and related adult diseases [18–20].

At present, many studies have been conducted to elucidate the correlation between IL-4-590C > T gene polymorphism and the susceptibility to asthma [18–20]. At the same time, some studies have shown that the IL-4-590C > T TT genotype has a higher susceptibility to asthma than the IL-4-590C > T CC genotype. However, these results are still inconsistent [18–20]. Therefore, this meta-analysis included the relative literature about the interplay between the polymorphism of IL-4-590C > T and the susceptibility to asthma and further explored the specific impact of polymorphism of IL-4-590C > T in the development of asthma.

## 2. Materials and Methods

### 2.1. Literature Search

This meta-analysis mainly searched for the included case-control studies or cohort studies on the relationship between the polymorphism of IL-4-590C > T and the susceptibility to asthma. The online databases Embase, PubMed, and Cochrane Library were systematically searched until June 2019. The search terms included the following: “Interleukin-4” or “IL-4-590C > T,” “single nucleotide polymorphism” or “variants,” or “polymorphism” and “asthma,” and “risk” or “susceptibility”. In addition, some of the selected references in this meta-analysis were manually searched so as to include potentially eligible literature. The two researchers independently screened the literature that might meet the inclusion criteria independently through the retrieved literature titles and abstracts and further determined whether to include them based on the full text. The authors used the combination of online search and manual search to avoid missing the literature. After cross-checking, the disputed data were discussed. If there were the same data or overlapping data, the largest or most recently published study was included.

### 2.2. Inclusion Criteria

The inclusion criteria were limited to all published articles, and a case-control/cohort study about the association between IL-4-590C > T and susceptibility to asthma was selected. Inclusion criteria were as follows: (1) a cohort study or case-control study; (2) the relationship between the risk of asthma and IL-4-590C > T gene polymorphism was reported; (3) the odds ratio (OR) and 95% confidence interval (CI) of the literature were provided. Exclusion criteria were as follows: (1) a cross-sectional study or case report study; (2) the literature that assesses only asthma was excluded; (3) the study that provided only the ORs without providing 95% CI. In addition, the documents of repeated reporting or poor quality were also not included in the review or abstract literature.

### 2.3. Data Extraction

Baseline data were extracted including first author, age, ethnicity, source of controls, genotyping methods, sample size, the related confounding factors, and ORs and 95% CI about IL-4-590C > T gene polymorphism and asthma risk. According to the data table set up by the research institute, two researchers independently extracted the data and then cross-checked. Subsequently, any disagreement should be discussed with the third reviewer until the agreement was reached.

### 2.4. Statistical Analysis

The ORs and the corresponding 95% CI on the association between IL-4-590C > T polymorphism and susceptibility of asthma were extracted from included articles using the raw data. The fixed-effect model (the Mantel–Haenszel method) and the random effects model (the DerSimonians–Laird method) were used in the meta-analysis. If the *PP* value is less than 0.05, the random effects model was used; otherwise, the fixed-effects model was performed in this meta-analysis. The process of meta-analysis first evaluated the statistical heterogeneity between the combined studies and then performed a combined analysis. In addition, subgroup analysis was further conducted based on ethnicity, source of controls, and genotyping methods to explore potential sources of heterogeneity. Sensitivity analysis reflected the stability and reliability of the results by excluding individual studies item by item and recalculating their ORs. Publication bias was evaluated by depicting Begg's funnel plots and applying for Egger's linear regression test. Besides, *P* < 0.05 was considered as statistically significant. Statistical analysis was performed by STATA software (version 12.0).

## 3. Results

### 3.1. Characteristics of the Studies

In the current meta-analysis, 818 asthma patients and 831 healthy individuals participated in these 8 independent case-control studies [18, 19, 21–25]. In Table 1, the genotype distribution and detailed characteristics of the selected studies about the relationship between the polymorphism of IL-4-590C > T and the susceptibility to asthma are displayed.  Figure 1 shows the literature search and selection process, as well as a description of the reasons. In the included studies, three studies were conducted on Caucasians and the others were on Asians. In addition, to distinguish the source of control, we also conducted subgroup analysis based on the population-based control group and the hospital-based control group. In addition, different genotyping methods included TaqMan and PCR-RFLP.

### 3.2. Quantitative Synthesis Results

Totally, the primary outcome of meta-analysis of the relationship between the IL-4-590C > T polymorphism and the susceptibility to asthma was as follows: initially, the results showed no significant relationship between the TT genotype of IL-4-590C > T and the increased susceptibility to asthma in the random effects model (dominant model: OR = 1.31, 95% CI = 0.68–2.53) (Figure 2).

Subgroup analyses were performed based on ethnicity, source of control, and genotyping methods to evaluate the effect of heterogeneity on the results. Subgroup analysis by ethnicity revealed no significant results in the Asian population (OR = 1.28, 95% CI = 0.24–6.80); however, the TT genotype of IL-4-590C > T significantly increased the susceptibility to asthma in the Caucasian population (OR = 1.43, 95%CI = 1.03–1.98) (Figure 3(a)). Subgroup analysis by source of control was performed. A statistically significant result was found in the population-based control group (OR = 1.33, 95% CI = 1.01–1.76), but not in the hospital-based control group (OR = 1.22, 95% CI = 0.27–5.46) (Figure 3(b)). Additionally, subgroup analysis was performed by genotyping methods and no significant statistics were found in the PCR (OR = 1.21, 95% CI = 0.37–3.96) and the TaqMan (OR = 1.58, 95% CI = 0.95–2.63) (Figure 3(c)).

### 3.3. Sensitivity Analysis

Sensitivity analysis was conducted by omitting individual studies one by one, and the effect of each individual study on recalculating ORs was examined by repeated meta-analysis.  Figure 4 shows sensitivity analysis on the polymorphism of IL-4-590C > T gene and the risk of asthma, indicating that the combined ORs have no significant effect. Therefore, sensitivity analysis indicated that the results of this meta-analysis were reliable.

### 3.4. Publication Bias

Begg's funnel plot and Egger's test were used to assess the publication bias of this meta-analysis. The results found that the shape of the funnel plot appeared to be symmetrically distributed, indicating that no publication bias was found in the meta-analysis (Begg's test: *P* = 0.999; Egger's test: *P* = 0.589) (Figure 5).

## 4. Discussion

At present, most researchers suggested that asthma might be caused by many different genes. Previous studies have found that the occurrence of asthma has strong genetic characteristics, with a heritability of up to 60%–80%. However, it does not fully comply with the classical Mendelian inheritance law, which is often caused by the interaction of multiple genetic and environmental factors and other susceptibility factors [8–10]. Most studies have shown that cytokines affect the type and duration of inflammatory response in patients with asthma caused by various causes and play an important role in the transmission between various inflammatory cells [5–7]. Because of various external reasons, the inflammatory response with different inflammatory mediators interacted with each other to increase the reactivity of the airway and produced inflammation and aggravation in the airway, leading to the occurrence of asthma [3, 7–9]. IL-4, as a representative of inflammatory mediators during the development of asthma, might be stimulated in the body, and the initial part of IgE synthesis played a vital part in the level of IgE in plasma [13–16]. In this meta-analysis, the relationship between different bases on multiple gene loci and the occurrence of asthma was investigated to explore whether the mutation of bases on IL-4 gene loci has certain interaction with the susceptibility of asthma [17, 18].

Many scholars have conducted a series of studies on related genes, with different results, which explored whether the polymorphism of IL-4 was correlated with the risk of asthma [18, 20]. Therefore, the polymorphism of IL-4-590C > T gene in the risk of asthma has not been clearly concluded. The study of Hussein et al. [21] showed that the increased susceptibility to asthma was associated with the C allele and CC genotype of IL-4-590C > T gene polymorphism, which was considered to be the etiological part of asthma. However, it was found that the higher the percentage of T allele in the control group, the lower the susceptibility to asthma [18, 19, 21–24]. Another study by Zhang et al. [18] suggested that the polymorphism of IL-4-590C > T was associated with the bronchial asthma in Uyghur children, and the T allele might be a risk factor in Uyghurs. In addition, the variant in this gene could lead to increased IgE levels and decreased FEV1 levels, indicating that they were related with bronchial asthma in Uyghur children [18]. However, there is no consistent conclusion about the polymorphism of IL-4-590C > T and the risk of asthma. In this meta-analysis, we attempted to elucidate whether the gene polymorphism of IL-4-590C > T was associated with the susceptibility to asthma.

In recent years, the research studies on asthma-related genes have been developing. This meta-analysis has made better understanding about the association between the gene polymorphism of IL-4-590C > T and the risk of asthma by different subgroup analyses. Therefore, a meta-analysis was used to elucidate this possible association. In this meta-analysis, 6 independent case-control studies included 818 asthmatic patients and 831 healthy individuals. The results showed no significance between the gene polymorphism of IL-4-590C > T and increased susceptibility to asthma. The results might be due to different sample size, genotyping methods, study design, statistical methods, and other factors. Subsequently, in subgroup analyses by ethnicity, no statistically significant correlation was observed based on the Asian population. However, the polymorphisms in the IL-4-590C > T gene were found to increase the susceptibility to asthma in Caucasian. Besides, subgroup analysis was performed by source of control. A statistically significant result was found in the population-based control group, but not in the hospital-based control group. In subgroup analysis based on genotyping methods, no statistical significance was observed for this correlation, whether based on PCR and TaqMan.

In summary, the pathogenesis of asthma is still not very clear and the induction and participation in the pathogenesis of asthma are also coaffected by environmental, genetic, endocrine, and other factors [10–12]. Asthma is a disease in which many different genes are involved. A single disease-causing gene might have a weak effect on the occurrence of asthma. Therefore, in the subsequent years, we need to conduct more in-depth research on the effect of different asthma-related genes and whether there was synergy between multiple genes on the occurrence of asthma, which might provide a more accurate treatment for asthma [11]. In this meta-analysis, the polymorphism of IL-4-590C > T gene was studied to understand the susceptibility of asthma, and the IL-4 gene site mutation had a synergistic effect on the development of asthma.

However, this meta-analysis has certain limitations. Considering that the number of specimens that could be used for research was small, there might be partial false negative results, and there is no stratification of the degree of asthma at the beginning of the study. Therefore, future research needs to increase the sample size and further analyze the severity of asthma. The pathogenesis of asthma is complex. Whether IL-4 gene polymorphism is correlated with the pathogenesis of asthma or not needs further study. Only studying asthma-related genes could better discuss the pathogenesis of asthma and provide theoretical basis for the prevention and treatment of asthma.

## 5. Conclusions

This meta-analysis indicated that the TT genotype of the gene polymorphism of IL-4-590C > T significantly enhanced the susceptibility to asthma in Caucasian populations, but not in Asian populations. In addition, because of the limitations of the quantity and quality of included studies, more prospective studies with large samples were needed for further confirmation.

## Figures and Tables

**Figure 1:** Flow diagram of searching and selection process of the eligible literature.

**Figure 2:** Forest plots depicted based on the association between IL-4-590C > T polymorphism and susceptibility to asthma in the dominant model.

**Figure 3:** Forest plots depicted based on subgroup analysis of the association between IL-4-590C > T polymorphism and susceptibility to asthma in the dominant model. Subgroup analysis based on (a) ethnicity, (b) source of controls, and (c) genotyping methods.

**Figure 4:** Sensitivity analysis in the random effects model.

**Figure 5:** Begg's funnel plots depicted for the publication bias test.

**Table 1:** Characteristics of studies that investigated the association between interleukin-4-590C > T polymorphism and the risk of asthma.

Author	Year	Country	Ethnicity	SOC	Genotyping methods	No. of cases	No. of controls	Case (*N*)			Control (*N*)			HWE
								CC	CT	TT	CC	CT	TT	
Zhang	2019	China	Asian	PB	PCR	37	29	7	13	17	11	15	3	Y
Hussein	2017	Iraq	Asian	HB	PCR	48	25	42	5	1	8	13	4	Y
Zhang	2016	China	Asian	HB	PCR	38	35	8	11	19	17	13	5	Y
Berenguer	2014	Portugal	Caucasian	HB	TaqMan	98	105	63	32	3	84	20	1	Y
Smolnikova	2013	Russia	Caucasian	PB	PCR	128	50	72	50	6	30	19	1	Y
Amirzargar	2009	Iran	Asian	HB	PCR	58	139	0	59	0	10	129	0	N
Adjers	2005	Finland	Caucasian	PB	TaqMan	243	401	99	144	189		212		Y
Hijazi	2000	Kuwait	Asian	HB	PCR	84	47	5	25	54	3	17	27	Y

SOC, source of controls; PB, population-based controls; HB, hospital-based controls; HWE, Hardy–Weinberg equilibrium.

## Data Availability

The datasets used and analyzed during the current study are available from the corresponding author on reasonable request.
